# *BRAF* Testing in Multifocal Papillary Thyroid Carcinoma

**DOI:** 10.1155/2015/486391

**Published:** 2015-09-13

**Authors:** Hillary Z. Kimbrell, Andrew B. Sholl, Swarnamala Ratnayaka, Shanker Japa, Michelle Lacey, Gandahari Carpio, Parisha Bhatia, Emad Kandil

**Affiliations:** ^1^Department of Pathology and Laboratory Medicine, Tulane University, 1430 Tulane Avenue SL-79, New Orleans, LA 70112, USA; ^2^Department of Mathematics, Tulane University, 6823 St. Charles Avenue, New Orleans, LA 70118, USA; ^3^Department of Medicine, Tulane University, 1430 Tulane Avenue SL-12, New Orleans, LA 70112, USA; ^4^Department of Surgery, Tulane University, 1430 Tulane Avenue SL-22, New Orleans, LA 70112, USA

## Abstract

*Background. BRAF* V600E mutation is associated with poor prognosis in patients with papillary thyroid carcinoma (PTC). PTC is often multifocal, and there are no guidelines on how many tumors to test for *BRAF* mutation in multifocal PTC. *Methods*. Fifty-seven separate formalin-fixed and paraffin-embedded PTCs from twenty-seven patients were manually macrodissected and tested for *BRAF* mutation using a commercial allele-specific real-time polymerase chain reaction-based assay (Entrogen, Woodland Hills, CA). Data related to histologic characteristics, patient demographics, and clinical outcomes were collected. *Results*. All mutations detected were *BRAF* V600E. Seventeen patients (63%) had concordant mutation status in the largest and second-largest tumors (i.e., both were positive or both were negative). The remaining ten patients (37%) had discordant mutation status. Six of the patients with discordant tumors (22% overall) had a *BRAF*-negative largest tumor and a *BRAF*-positive second-largest tumor. No histologic feature was found to help predict which cases would be discordant. *Conclusions*. Patients with multifocal PTC whose largest tumor is *BRAF*-negative can have smaller tumors that are *BRAF*-positive. Therefore, molecular testing of more than just the dominant tumor should be considered. Future studies are warranted to establish whether finding a *BRAF* mutation in a smaller tumor has clinical significance.

## 1. Introduction

Papillary thyroid carcinoma (PTC) is often a multifocal disease, with rates as high as 80% in the literature [1]. Despite multiple studies using different methodologies [1–11] it remains an unsettled question as to whether the multifocality represents separate primary tumors or intraglandular metastasis, or a combination of both. It seems likely from prior studies that a subset of cases represent separate primaries, or at the very least have molecularly distinct tumors. The question then arises, how many tumors should be tested for* BRAF* mutation in multifocal PTC? A recent very large retrospective study found that patients with multifocal disease and a* BRAF* V600E mutation had a significantly higher rate of mortality than patients with multifocal disease without a* BRAF* mutation, but the study did not elaborate on how many or which tumors were tested for each patient [12]. Our study attempts to further the data on* BRAF* mutation status in patients with multifocal disease and to find the optimal strategy for* BRAF* testing in these patients.

## 2. Materials and Methods

The study protocol was approved by the IRB at Tulane University. The laboratory information system was searched for cases of multifocal papillary thyroid carcinoma in patients with all thyroid tissue removed, either as a single surgery or two separate surgeries, since January 1, 2006. Thirty-three cases were identified, and the slides from each case were reviewed by the study pathologists (H.Z.K. and A.B.S.). In all but one case, the entire thyroid was submitted. The following histologic features were recorded for each tumor: size, laterality, histologic variant, and the presence or absence of additional features such as irregular border, location close to the capsule, extrathyroidal extension, satellite nodules, and isolated psammoma bodies. Satellite nodules were defined as tumor foci less than 0.5 mm that were within one section of a larger tumor nodule but not directly attached to the larger nodule. Isolated psammoma bodies were defined as psammoma bodies within the thyroid parenchyma and separate from any tumor nodules. The histologic variant was decided by each pathologist separately, based on the predominant pattern seen in the tumor; discrepancies were resolved by viewing the case together at a multiheaded scope.

The study pathologists marked the two largest tumors in each case, and the tissue was manually macrodissected and placed into tubes. DNA was extracted using the EZ1 DNA Tissue kit (Qiagen, Valencia, CA).* BRAF* mutational status was tested using a commercial allele-specific real-time polymerase chain reaction-based assay that can detect five point mutations in codon 600 (V600E, V600K, V600R, V600D, and V600M) when present in as little as 1% of the tissue (Entrogen, Woodland Hills, CA). Overall, six of the original thirty-three cases were excluded because of insufficient DNA (either a tumor focus was gone on deeper levels or the DNA was of poor quality), leaving a total of twenty-seven cases for the study (see Table 1). Two of the cases where both the largest and second-largest tumors were* BRAF*-negative had additional tumors (see Patients 24 and 25 in Table 1); three of these additional tumors had adequate DNA and were tested for* BRAF* mutation (two additional tumors for Patient 24 and one additional tumor for Patient 25). In all, a total of fifty-seven tumors were tested for* BRAF* mutation. Clinical data related to patient demographics, tumor stage, months of followup, and outcome was collected for these twenty-seven patients. Statistical calculations were performed using *R*, with the Student's *t*-test and Fisher's exact test used to calculate significance. To assess whether* BRAF* status was associated with positive lymph nodes independently of size, multivariate analysis was carried out using logistic regression and the corresponding likelihood ratio test. Additionally, a model was made to predict the size of each tumor (on the log scale) as a function of* BRAF* status and size.

## 3. Results

There were 17 women and 10 men included in the study with an average age at diagnosis of 52 (range: 26 to 78). The average number of tumor nodules rounded to the nearest whole number was 3, ranging from 2 to 9. Overall, 34 of the 57 tumors (60%) were* BRAF*-positive and all mutations were V600E.  Figure 1 illustrates the histologic variants and their respective rates of* BRAF* mutation. Notably, the tall cell variant had the highest rate of positivity for* BRAF* mutation (3 of 3 cases), and the encapsulated follicular variant had the lowest rate (1 of 6 cases). The one* BRAF*-positive encapsulated follicular variant showed focal invasion through the capsule and therefore should probably have been considered along with the other follicular variant tumors that showed an infiltrative growth pattern, as in Walts et al. [13]. There was no significant correlation between* BRAF*-positivity and the presence of an irregular border (*P* = 0.6), location close to the capsule (*P* = 0.8), or extrathyroidal extension (*P* = 1).

The overall average size of the largest nodule was 1.6 cm, ranging from 0.2 cm to 3.6 cm. There was no significant difference in size between the* BRAF*-negative and* BRAF*-positive largest nodules (average sizes 1.8 cm and 1.5 cm, *P* = 0.3). The overall average size of the second-largest nodule was 0.5 cm, ranging from 0.1 cm to 2.2 cm. There was no significant difference in size between the* BRAF*-negative and* BRAF*-positive second-largest nodules (average sizes 0.5 cm and 0.6 cm, *P* = 0.7).

A mutation was present in at least 1 nodule in 22 of the 27 cases (81.4%). In 17 patients, both the largest and second-largest nodules had concordant* BRAF* status; that is, they were both either positive or negative. The remaining ten patients had discordant mutation status; that is, one tumor was positive and one tumor was negative. No histologic features were significantly different between the concordant and discordant cases. The tumors were of the same histologic variant in 11 (65%) of the concordant cases, compared with 7 (70%) of the discordant cases (*P* = 1), as illustrated in Figure 2. Satellite nodules were present in 53% of the concordant cases and 20% of the discordant cases (*P* = 0.1). Isolated psammoma bodies were present in 41% of the concordant cases and 20% of the discordant cases (*P* = 0.4). The largest tumor had irregular borders in 65% of concordant cases and 70% of discordant cases (*P* = 1). Both the largest and second-largest tumors had smooth borders in 12% of the concordant cases and 10% of the discordant cases (*P* = 1).

Similarly, there was no significant correlation between concordant mutation status and laterality: the largest and second-largest tumors were in the same lobe in 6 of the 17 concordant cases (35%), compared to 2 of the 10 discordant cases (20%, *P* = 0.7). The two largest tumors were concordant in 4 of the 5 cases where the disease was unilateral (80%), compared to 13 of the 22 cases that were bilateral (59%, *P* = 0.6).

Cases with 4 or more nodules tended to have concordant mutation status (8 of 9, or 89%) compared to cases with fewer than 4 nodules (9 of 18, or 50%) but this did not reach statistical significance (*P* = 0.09).

Lymph node dissection was performed at the discretion of the surgeon (E.K.) who was not aware of the* BRAF* status preoperatively. There was a significant difference in nodal stage between the patients with a* BRAF*-positive largest tumor and a* BRAF*-negative largest tumor: 11 of the 16 patients (69%) with a* BRAF*-positive largest tumor had cervical lymph node metastases (either N1a or N1b) compared to 2 of the 11 patients (18%) with a* BRAF*-negative largest tumor (*P* = 0.02). This association remained significant when a multivariate analysis was done to account for tumor size (*P* = 0.005). With regards to the largest tumors, the smallest of these were the* BRAF*-negative tumors with positive lymph nodes (*P* = 0.04), followed by the* BRAF*-positive tumors with negative lymph nodes (*P* = 0.06). There was no significant size difference between the* BRAF*-negative tumors with negative lymph nodes and the* BRAF*-positive tumors with positive lymph nodes. Of note, none of the six patients with a* BRAF*-negative largest tumor and* BRAF*-positive second-largest tumor had positive lymph nodes.

None of the patients presented with or experienced distant metastases. Overall, the average amount of clinical followup was 20 months (range <1 month to 81 months). Two of the 27 patients (7.4%) had recurrence in the cervical lymph nodes, one at 7 months postsurgery/3 months post-radioactive iodine and one at 19 months postsurgery/16 months post-radioactive iodine. These two patients were* BRAF*-positive in both the largest and the second-largest tumors. None of the remaining patients had a definitive recurrence. One patient with a* BRAF*-negative largest tumor and a* BRAF*-positive second-largest tumor did have positive radioactive iodine uptake in the mediastinum after surgery, but it was unclear whether this represented ectopic thyroid tissue or recurrent disease and the area was not amenable to biopsy.

## 4. Discussion

In this study, we attempted to find the optimal approach for* BRAF* mutation testing in multifocal PTC. One hypothetical strategy would be to test each tumor sequentially, starting with the largest tumor and working towards the smallest until a mutation is found; however, this would require strong coordination between the surgical pathologist and molecular pathologist and would not be the most timely or cost-effective strategy, given that each tumor would be tested on a separate run. At the other extreme, another strategy would be to test all of the tumors up front, but since twelve of our patients (44%) had three or more tumors, testing every single nodule may be costly with overuse of resources. We sought an approach somewhere in between these two extremes.

Not surprisingly, all of our tall cell variants were* BRAF*-positive, which is consistent with the generally accepted idea that tall cell variant has the highest rate of* BRAF* positivity (around 80% [14]). This indicates that tumors with tall cell histology should be prioritized in any testing algorithm.

The follicular variant had the lowest rate of* BRAF*-positivity at 42%. This percentage is high relative to the generally accepted value of around 10% [14], but is in line with more recent studies that used more sensitive molecular techniques and found* BRAF*-positivity in 21% to 54% of follicular variants [13, 15–17]. Additionally, in the current study, three of the follicular variants that were positive were in the same gland as a* BRAF*-positive classic variant (see Table 1) and therefore could have been intraglandular metastases. Walts et al. specifically excluded cases like this from their study of follicular variants and were very strict on the definition of follicular variant (requiring 95% or more of the tumor to have follicular architecture); their study had a rate of 33.3%* BRAF*-positivity (16 of 48 cases, which included both unifocal and multifocal cases) [13]. Therefore, follicular variant tumors should not be excluded from the testing algorithm, with the caveat that tumors that are completely encapsulated have a very low chance of being positive.

In this study, 10 cases (37%) had tumors with discordant* BRAF* mutation status. This is in line with other studies that have reported discordant* BRAF* mutation status in 14% to 39% of multifocal PTC cases [2, 3, 8, 10, 11]. Ideally, there would be some histologic feature to help identify which cases are likely to have discordant mutation status and therefore indicate that more than just the largest tumor should be tested. We first looked at whether discordant tumors tended to be of different histologic variants because in Park et al. tumors were of different histologic variants in 58.3% of discordant cases compared to 32.4% of concordant cases (*P* = 0.047) [8]; similar observations were made by Bansal et al. [1] and Giannini et al. [2]. We did not find this in our study, however, as discordant tumors were statistically equally likely to be of the same or different histologic variants.

Another variable we examined was whether concordant tumors were more often in the same lobe. In Bansal et al., tumors with the same mutation (*BRAF*,* RAS,* or* RET/PTC*) were statistically more likely to be in the same lobe when compared to those with different mutations (60% versus 22.2%, *P* = 0.04) [1]. Similarly, Kuhn et al. found that tumors with concordant X chromosome inactivation patterns tended to be in the same lobe and discordant tumors were in contralateral lobes [4]. However, Park et al. did not find a correlation between* BRAF* mutation concordance and laterality: 9 of 24 unilateral cases (37.5%) had mixed* BRAF* status compared to 15 of 37 bilateral cases (40.5%, *P* > 0.05) [8]. Our findings were similar to Park et al. in that tumors with concordant mutations were not more likely to be in the same lobe, and tumors with discordant mutations were not more likely to be in opposite lobes.

We next examined whether the presence of satellite nodules indicated a concordant mutation status. In theory, satellite nodules should result from intraglandular metastasis and therefore all tumors would have the same mutational status. In Bansal et al., microscopic peritumoral dissemination (which is similar to what we are calling satellite nodules) was seen at a significantly lower rate in cases with different mutations (*P* = 0.029) [1]. We found a similar trend: cases with satellite tumors did tend to have concordant mutation status, but this did not reach statistical significance. Isolated psammoma bodies, which again should indicate intraglandular metastasis, also did not correlate significantly with concordant mutation status.

Bansal et al. noted that >60% of tumors with different mutations had smooth borders, with the idea that a smooth border indicates a less aggressive tumor that would be unlikely to develop intraglandular metastasis. In other words, multiple tumors with smooth borders would more likely represent separate primaries, and tumors with irregular borders would more likely represent intraglandular metastasis [1]. We did not find any significant association between smooth borders and discordant mutation status, or irregular borders and concordant mutation status, however.

Cases with more than three tumor foci were more likely to have discordant* BRAF* status in Park et al. [8], but our study found a trend in the opposite direction: cases with more nodules tended to be concordant, but this did not reach statistical significance.

In summary, there does not seem to be a reliable way to predict which cases will have tumors with discordant* BRAF* status. However, from our limited data it does seem that testing more than two tumors may not be necessary: of the five cases where the two largest tumors were both negative, two cases had additional nodules with adequate DNA for testing, and these three additional nodules were all* BRAF*-negative. In other words, although our numbers were limited, we did not find any cases where a third-largest or fourth-largest tumor was* BRAF*-positive when the largest and second-largest tumors were* BRAF*-negative.

Importantly, six of our cases (22%) had a* BRAF* mutation in the second-largest tumor when the largest tumor was* BRAF*-negative. This is similar to Ahn et al., where thirteen out of eighty-five patients with multifocal PTC (15%) had a* BRAF* mutation in a smaller nodule when the largest was* BRAF*-negative [18]. Therefore, if only the largest tumor is tested, a substantial number of patients would be considered* BRAF*-negative even though they harbor a smaller tumor that is* BRAF*-positive.

The clinical significance of finding a* BRAF* mutation in a nondominant tumor, however, is unknown. Among our cohort, none of the six patients with a* BRAF*-negative largest tumor and* BRAF*-positive second-largest tumor presented with positive lymph nodes or had a definitive recurrence, although one patient had a small area of positivity on a radioiodine scan that was either a positive mediastinal lymph node or ectopic thyroid tissue (the area was not amenable to biopsy and the patient was given adjuvant radioiodine). Our study is too small and the followup is too short to draw further conclusions, but the two patients who experienced a definite recurrence had a* BRAF* mutation in both their largest and second-largest nodules. This finding is of interest, since Ahn et al. found that the patients who were* BRAF*-positive in all of their nodules had significantly higher rates of extrathyroidal invasion, lymph node metastases, and postoperative radioactive iodine therapy, when compared to the group with mixed mutation status. Thus, having a* BRAF* mutation in all nodules likely indicates more aggressive disease, probably because the tumors represent intraglandular spread from the same primary [18].

We note that this study had a relatively high rate of* BRAF* mutation (42% of the follicular variants, as described above, and 60% of the tumors overall), which may be due to two factors: first,* BRAF* mutation may be more frequent in multifocal disease [18, 19] and second, our* BRAF* assay has high analytic sensitivity. Recent studies have found that* BRAF* mutation is most likely not present in every cell of a given tumor and that the percentage of mutated alleles may vary regionally within the tumor. Thus, an assay that can detect a smaller percentage of mutated alleles will call more tumors positive [20–24]. One excellent example of how analytic sensitivity can affect the rate of* BRAF* mutations is seen in Guerra et al., who used two different assays in their study: BigDye Terminator sequencing (PE Applied Biosystems, Foster City, CA) and pyrosequencing. By BigDye Terminator sequencing,* BRAF* mutation was identified in 62 of 168 (36.9%) cases of unifocal papillary thyroid carcinoma and by pyrosequencing, it was identified in 90 of 168 (53.6%). This resulted in differences in the clinical variables that were significantly associated with the presence of* BRAF* mutation. For example, lymph node metastasis and AJCC stage I disease had positive associations with* BRAF* mutation by BigDye Terminator sequencing (*P* = 0.012 and *P* = 0.016, resp.) but neither had significant associations by pyrosequencing. Recurrence was 2.1 times more likely in* BRAF*-positive patients by BigDye Terminator sequencing (*P* = 0.040), but there was no significant difference in recurrence by pyrosequencing [24]. Clearly, the choice of assay can affect both the rate of* BRAF* mutation and its clinical utility. This means that the results from our study may not be generalizable to labs that use a less sensitive assay.

We also note that the study cohort contained a high number of male patients (10 out of 27, or 37%). One possibility for this is that the percentage of men might be higher among patients with multifocal disease as was found in Huang et al. [25], who studied 648 patients with PTC in China. In their study, 49 of 168 patients with multifocal disease were male (29%) compared to 89 of 480 patients with unifocal disease (19%, *P* = 0.004). However, other studies have found nearly equal percentages of males in both multifocal and unifocal cases, ranging from 16% to 24% [11, 26, 27]. Therefore, it is more likely that the high number of male patients reflects some bias in the types of patients referred to the study surgeon. Since the percentage of cases with discordant* BRAF* mutations is in line with previous studies, as discussed above, it is unlikely that this bias had a great effect on our results.

## 5. Conclusions

Patients with multifocal PTC whose largest tumor is* BRAF*-negative can have smaller tumors that are* BRAF*-positive. Therefore, molecular testing of more than just the dominant nodule should be considered, especially if a smaller tumor has tall cell features. Future larger studies are warranted to establish whether finding a* BRAF* mutation in a smaller tumor correlates with more aggressive disease.

## Figures and Tables

**Figure 1:** Histologic variants and rates of* BRAF* mutation. The percentage given after the number of cases indicates the rate of* BRAF* mutation for that particular variant. Follicular variant is broken down into encapsulated and nonencapsulated.

**Figure 2:** Breakdown of cases relative to mutation concordance and histologic variant(s) of the largest and second-largest tumors. The number in parentheses indicates the number of cases. Clas = classic variant, Fol = follicular variant, TC = tall cell variant, War = Warthin-like variant, Onc = oncocytic variant, and ∗ = one patient in this subgroup experienced a recurrence.

**Table 1:** Patient characteristics.

Patient number	Age	Sex	Months of Followup	Initial pTN	Number of nodules	Size of largest nodule (cm)	Histologic variant of largest nodule	BRAF status of largest nodule	Size of second-largest nodule (cm)	Histologic variant of second-largest nodule	BRAF status of second-largest nodule
1	40	F	34	T1b N1a	4	1.4	Fol	Positive	0.8	Fol	Positive
2	64	M	40	T3 N1b	2	1.2	TC	Positive	0.5	Clas	Positive
3	74	M	1	T3 N1b	4	1.1	Clas	Positive	0.3	Clas	Positive
4^*^	58	M	13	T3 N1b	2	1.3	Clas	Positive	0.4	Fol	Positive
5	65	M	2	T1a N1a	5	1.0	Clas	Positive	0.9	Clas	Positive
6	78	M	9	T1a N0	4	0.5	Clas	Positive	0.2	Clas	Positive
7	55	F	29	T2 N0	6	2.5	TC	Positive	0.4	War	Positive
8	59	F	4	T1b N1b	2	1.5	Fol	Positive	0.2	Fol	Positive
9^*^	50	M	50	T1a N0	3	0.9	Clas	Positive	0.8	Clas	Positive
10	28	F	6	T3 N1a	8	2.2	Clas	Positive	2.2	Clas	Positive
11	63	M	3	T1b N1a	2	1.2	Clas	Positive	0.2	Fol	Positive
12	26	F	3	T1b N1a	2	1.4	Clas	Positive	0.3	Fol	Positive
13	43	M	23	T2 N1b	3	3.6	TC	Positive	0.2	Fol	Negative
14	50	F	22	T3 N0	3	0.4	Clas	Positive	0.1	Fol	Negative
15	42	F	22	T2 N1a	2	2.6	Clas	Positive	0.2	Clas	Negative
16	44	F	11	T1a N0	2	0.7	Onc	Positive	0.4	Onc	Negative
17	37	F	10	T1a N0	2	1.0	Clas	Negative	0.3	Clas	Positive
18	45	F	8	T2 N0	9	2.4	Fol	Negative	0.5	Fol	Positive
19^‡^	49	F	56	T2 N0	2	2.4	Fol	Negative	0.6	Fol	Positive
20	53	M	6	T2 N0	2	2.4	Fol	Negative	0.2	Fol	Positive
21	49	F	20	T1a N0	2	0.2	Fol	Negative	0.1	Fol	Positive
22	76	F	1	T3 N0	2	1.2	Fol	Negative	0.9	Clas	Positive
23	53	F	79	T3 N0	2	2.0	Fol	Negative	2.0	Fol	Negative
24^**^	32	F	4	T1b N1b	4	2.0	Clas	Negative	0.2	Clas	Negative
25^**^	67	F	<1	T1b N1a	5	1.1	Onc	Negative	0.2	Fol	Negative
26	48	F	81	T2 N0	2	3.5	Fol	Negative	0.7	Fol	Negative
27	60	M	<1	T1b N0	2	1.9	Fol	Negative	0.5	Fol	Negative

The ∗ indicates that the patient experienced a recurrence (Patient 4 at 7 months postsurgery/3 months post-radioactive iodine and Patient 9 at 19 months postsurgery/16 months post-radioactive iodine). The ‡ indicates a patient who had a possible recurrence that could not be biopsied and was treated with radioiodine. The ∗∗ indicates that additional tumors were tested for these patients (Patient 24: two additional nodules, Patient 25: one additional nodule); the additional nodules were all negative. Fol = follicular variant, TC = tall cell variant, Clas = classic variant, Onc = oncocytic variant, War = Warthin-like variant.
